RETRACTED

# RNF43 ubiquitinates and degrades phosphorylated E-cadherin by c-Src to facilitate epithelial-mesenchymal transition in lung adenocarcinoma

**DOI:** 10.1186/s12885-019-5880-1

**Published:** 2019-07-08

**Authors:** Yunfeng Zhang, Liangzhang Sun, Xiao Gao, Aining Guo, Yan Diao, Yang Zhao

**Affiliations:** 1 Department of Oncology, the Second Affiliated Hospital of Xi’an Jiaotong University, Xi’an, Shaanxi Province People’s Republic of China 710004; 2 Thoracic Department, the Second Affiliated Hospital of Xi’an Jiaotong University, Xi’an, Shaanxi Province People’s Republic of China 710004; 3 Second Thoracic Department, the First Affiliated Hospital of Xi’an Jiaotong University, Xi’an, Shaanxi Province People’s Republic of China 710004

**Keywords:** RNF43, C-Src, Caspase-8, EMT

## Abstract

**Background:**

In epithelial cells, tyrosine kinases induce tyrosine phosphorylation and ubiquitination of the E-cadherin complex, which is responsible for the epithelial-mesenchymal transition (EMT). However, the precise mechanisms remain unclear.

**Methods:**

Protein antibody microarray analysis and E3 ligase profiling were performed to detect the unique E3 ligase underlying E-cadherin downregulation in lung adenocarcinoma tissues. Gene knockdown was performed using viral shRNA. Immunoblotting, immunofluorescence, immunoprecipitation, and xenograft models in vivo were integratively applied to explore RNF43-induced EMT in lung adenocarcinoma cell lines.

**Results:**

Protein antibody microarray analysis and E3 ligase profiling revealed that the RING finger protein 43 (RNF43) was linked to E-cadherin downregulation within the context of c-Src activation in lung adenocarcinoma tissues. In addition, the c-Src-Caspase-8 interaction markedly increased c-Src activity. Activated c-Src phosphorylated E-cadherin at the tyrosine 797 site to initiate RNF43-mediated E-cadherin ubiquitination at lysine 816 and subsequent degradation, thus allowing the nuclear translocation of β-catenin and upregulation of Vimentin and RNF43 expression in lung adenocarcinoma cells. Decreased E-cadherin expression and increased Vimentin expression induced the EMT phenotype and promoted tumor metastasis. The Frizzled 8 (Frz8)-RNF43-induced ubiquitination of phosphorylated E-cadherin was blocked by a monoclonal antibody against the cysteine-rich domain (CRD) of Frz8 but not by antibodies against the protease domain (PA) of RNF43.

**Conclusions:**

Our data suggest that RNF43 participates in the regulation of EMT in the metastasis of lung adenocarcinoma through the ubiquitination and degradation of phosphorylated E-cadherin by activated c-Src.

**Electronic supplementary material:**

The online version of this article (10.1186/s12885-019-5880-1) contains supplementary material, which is available to authorized users.

RETRACTED

## Background

Lung cancer has been the leading cause of cancer-related mortalities for decades and has a 5-year overall survival (OS) of 15% worldwide [1]. Furthermore, 80–85% of lung cancers are characterized as non-small cell lung cancer (NSCLC), with lung adenocarcinoma, which has a markedly increased incidence rate and a high death rate, being the most common subtype [1, 2]. Even if diagnosed at an early stage and surgically removed, lung adenocarcinoma can reoccur within months, spreading to the regional or distant lymph nodes, contralateral lung, and distant organs [2, 3]. Metastasis is an ominous feature of lung adenocarcinoma and remains the cause of 90% of deaths due to lung adenocarcinoma [4]. Little is known about the genetic and molecular mechanism of metastasis despite its clinical significance.

Epithelial-mesenchymal transition (EMT) is a prometastatic process by which epithelial cells undergo morphological changes upon the downregulation of epithelial cell markers, such as E-cadherin, and the upregulation of mesenchymal cell markers, such as Vimentin [5–9]. Notably, the nuclear import of β-catenin plays an important role in the EMT process [8, 10, 11]. β-catenin translocates into the nucleus under the stimulation of the Wnt signal [10, 11]. Subsequently, nuclear β-catenin forms a complex with T-cell factor/lymphoid enhancer factor (TCF/LEF) to regulate the transcription of a plethora of target genes. A previous study revealed that activated c-Src exclusively tagged E-cadherin with phosphotyrosine under growth factor-induced stimulation [12, 13]. This event was followed by the ubiquitination and degradation of E-cadherin by an E3 ligase, called Hakai, to facilitate EMT through the nuclear import of β-catenin to form a transcriptional complex with TCF/LEF [12, 13]. We previously observed that the c-Src-Caspase-8 interaction efficiently overactivated c-Src to induce EMT [14], leading to the question of whether the c-Src-Caspase-8 interaction is sufficient to trigger the EMT phenotype through E-cadherin phosphorylation and degradation to free β-catenin to form a complex with TCF/LEF. Our current data showed that c-Src was efficiently activated in a Caspase-8-dependent manner in lung adenocarcinoma cells. In contrast, Hakai was expressed at a much lower level in lung adenocarcinomas, and a transmembrane E3 ubiquitin ligase, RNF43, was exclusively identified to be ubiquitously expressed and associated with reduced E-cadherin expression in lung adenocarcinomas. Furthermore, RNF43 was shown to ubiquitinate and degrade phosphorylated E-cadherin at the cytoplasmic tyrosine 797 site by c-Src, allowing EMT via the nuclear translocation and subsequent interaction of β-catenin with TCF-4. This process was shown to govern a wide variety of target genes, including Vimentin, and was efficiently abrogated by a monoclonal antibody against RNF43.

RETRACTED

## Methods

### Patients, protein extractions and protein microarrays

Protein microarray was performed as we previously described [14]. Paired lung adenocarcinoma and paracancerous tissues (**≥** 2.0 cm to primary tumor) were obtained from 60 lung adenocarcinoma patients after surgeries at the First and the Second Affiliated Hospital of Xi’an Jiaotong University (2007–2010). Two individual pathologists analyzed lung adenocarcinomas defined as the pathological stage I-IIIA according to the American Joint Committee on Cancer (AJCC) 2013. We regularly scheduled all eligible patients to a life-long follow-up at the intervals of three months during the first two years and at the intervals of six months for three more years. Once suspecting recurrent or metastatic events, radiological, endoscopic, and histological examinations were obligatory. Informed consent was obtained before the study. The study was approved by the ethics committee of Xi’an Jiaotong University. Laser capture microdissection was used to attain the purified cancerous or noncancerous compartments in the hematoxylin-eosin (HE) staining section. Simply, we extracted the proteins using a lysis buffer with 10.0 nmol/L Tris (pH 7.4), 1.0 mmol/L sodium orthovanadate, and 1.0% SDS. The lysates were heated, and sonicated for 10–30 s. The protein concentration was examined by the Protein Assay Kit (Bio-Rad, Hercules, CA). Protein extracts were iced on dry ice for analysis. A series of 620 monoclonal anti-mouse antibodies against E3 ubiquitin ligases were used to construct antibody-microarrays. Using a high precision robotic arrayer (Gene Machines, San Carlos, CA), the antibodies from Abcam were diluted and spotted on poly-L-lysine-coated glass slides (Telechem International Inc., Sunnyvale, CA) at 100 μg/ml with the volume of 1 μl. Every antibody was replicatively spotted twice on the chip.

We thawed and blocked the slides in PBS with 1% BSA (Sigma) and 0.5% Tween20 at room temperature for 1 h, with which protein extracts containing 400 μg of protein were incubated in a humidified chamber at the room temperature for 3 h. The slides were sequentially washed 3 times with high-salt PBS-T and low-salt PBS eahc for 10 min. Following the slides were dried by centrifugation at 500×g for 5 min, they were hybridized with a goat anti-mouse secondary antibody for 40 min. The chemiluminescence signals for each spot were captured using a microarray scanner (Axon Instruments Inc., Foster City, CA). Primary analysis was performed using the Genepix software package.

RETRACTED

### E-cadherin ubiquitination and degradation

Cells were cultured in the serum-starved condition for 1 day and plated onto 10 cm nontissue culture-treated dishes (1.0 × 10^6^ for one dish) precoated with 10 μg/ml Fibronectin (Millipore) for 2 days. The cells were lysed by 1% Triton-X100 lysis buffer involving 1% SDS to detect E-cadherin ubiquitination. Then, lysates were diluted 20-fold with 1% Triton-X100 lysis buffer before coimmunoprecipitation. Total cell lysates (TCLs) were used for immunoprecipitation using an anti-E-cadherin antibody (ab-1416 Abcam), in which ubiquitinated E-cadherin was detected by immunoblotting with an anti-ubiquitin antibody (ab-7780 Abcam).

### Protein delivery

The recombinant antibody 7A7 was delivered into A549 cells using the Chariot protein delivery kit. Briefly, 1 mg of protein was mixed with 6 ml of Chariot. The mixture was incubated at room temperature to allow complex formation. Next, the cells were washed with serum-free medium, and the Chariot-protein complex was added to the cells with an additional 400 ml of serum-free medium. The cells were then incubated at 37 °C for 2 h to allow protein internalization.

### Chromatin immunoprecipitation (ChIP) assay

ChIP assays were performed as reported previously [15]. Briefly, A549 cells were cross-linked with 1% formaldehyde at room temperature for 10 min and quenched with 0.4 mM glycine. Chromatin extracts were sheared by micrococcal nuclease digestion. The protein-DNA complexes were then immunoprecipitated with 3 mg of anti-TCF-4 monoclonal antibody or an anti-β-catenin monoclonal antibody bound to anti-mouse IgG-coated Dynabeads (Life Technologies). DNA was subjected to PCR with the following primer sets: RNF43-promoter: sense: 5′-TCAACTCTCTGGATAAGGTGGAATAGC-3′ and antisense: 5′-GACTTTTGGGGTGGGTGGGAAATA-3′; E-cadherin-promoter: sense: 5′-TCGGGCACCTGGCCAAGATACA-3′ and antisense: 5′-TGGACGCCCTGGCTTCTGAG-3′; and Vimentin promoter: sense 5′-GACAATGCGTCTCTGGCACGTCTT-3′ and antisense: 5′-TCCTCCGCCTCCTGCAGGTTCTT-3′. In addition, amplification of the c-Myc (MYC) enhancer was used as a positive control (sense: 5′-GCTCAGTCTTTGCCCCTTTGTGG-3′ and antisense: 5′-AACACCTTCCCGATTCCCAAGTG-3′).

### MALDI-mass

MALDI-Mass was performed according to a previous report [16]. E-cadherin was immunopurified from A549 cells and electrotransferred onto PVDF membranes. The E-cadherin band was excised from the membrane, which was then incubated with 100 mg/ml cyanogen bromide (CNBr, Sigma) in 70% formic acid for 2 days at room temperature. After washing with 23.5 L of water and drying, the resultant peptide mixture was resolved in 70 ml of water and analyzed by MALDI. To enrich phosphotyrosine-containing peptides, the CNBr digestion mixtures were purified using a Pi3 PhosphoTyrosine-QE Kit (Nest Group Inc.) and analyzed by mass spectrometry.

RETRACTED

### Mass spectrometric and bioinformatics analysis

Samples were concentrated to 100 μl, alkylated at room temperature for 30 min, desalted and further concentrated by chloroform:methanol precipitation. After precipitation, the pellet was resuspended in 20 μl of 25 mM ammonium bicarbonate containing 2 μg of trypsin (Promega, Madison, WI). A rapid in-solution microwave-assisted tryptic digestion was performed in a CEM discover microwave unit at 45 °C for 10 min. The reaction was quenched by the addition of 2 μl of 0.1% trifluoroacetic acid (TFA). We injected samples via an autosampler for separation by reversed-phase chromatography on a NanoAcquity UPLC system (Waters, Dublin, CA). Peptides were reloaded onto a precolumn (5 μm Symmetry BEH-130 C18, 180 × 20 mm) and separated on an analytical column (1.7 μm BEH-130 C18 column 100 × 100 mm, Waters, Dublin, CA) at a flow rate of 1 μl a minute and a gradient of 2% Solvent B to 90% Solvent B (where Solvent A is water + 0.1% formic acid and Solvent B is 100% acetonitrile + 0.1% formic acid) applied over 40 min with a total analysis time of 55 min. Peptides were eluted directly into a nanospray ionization source with a spray voltage of 2 kV and analyzed using an LTQ XL-Orbitrap mass spectrometer (Thermo Fisher, San Jose, CA). Precursor ions were analyzed in the FTMS at a 60,000 resolution. MS/MS was performed on the LTQ instrument operated in data-dependent mode, whereby the top 10 most abundant ions were subjected to fragmentation. Data were searched using the Mascot Search Algorithm (Matrix Sciences, London, UK).

### Spontaneous human xenograft metastasis

The spontaneous human xenograft metastasis experimental protocol was performed according to a previous study [14]. 4-week male BALB/c nude mice were obtained from the Shanghai Experimental Animal Center and kept at the laboratory animal center of Xi’an Jiaotong University. They were in line with the institutional Animal Care and Use Committee guidelines. Cells were cultured in fresh medium for 1 day and harvested; the cell concentration was modified to 3.0 × 10^7^/ml with 50% Matrigel (Sigma) in the serum-free RPMI-1640 medium. Next, 0.2 ml of the mixture was injected subcutaneously into the flank of each mouse. Tumors reaching approximately 300 mm^3^ after 2–3 weeks were surgically removed to ensure equal tumor burden. Xenograft growth was supervised (10/group) with monoclonal antibodies against RNF43 and Frz8 (25 mg/kg daily via oral gavage) starting 20 days after tumor implantation. Biweekly, mice were anesthetized with isofluorane (Janssen Pharmaceutica, Belgium), injected with n-luciferin (225 mg/g body weight, potassium salt, Xenogen Corp.), and imaged on the IVIS-100 bioluminescence imager (Xenogen Corp.). The organs, including the brain, liver, spleen, lung, kidney, and spinal column, were harvested in the mice exhibiting tumor-related death or 125 days after tumor xenograft removal. Then, the harvested organs were fixed in 4% paraformaldehyde overnight and analyzed by immunostaining to detect micrometastasis. As necessary, the mice were euthanized by cervical dislocation, quickly inducing unconsciousness. Experiments were performed in accordance with the national guidelines for the care and use of animals and guidelines of Xi’an Jiaotong University.

RETRACTED

### Statistical analysis

SPSS 16.0 software was used to perform the statistical analysis. The in vitro experiments were performed at least three times in triplicate. When comparing data among groups, normal analysis and homogeneity of variance were performed, followed by an unpaired two-tailed *t* test. Error bars on the graphs and the data in the text represent the mean ± SD. For in vivo studies, statistical power was determined by assessing all cohorts including experimental animals using the *χ*^*2*^ and Mann-Whitney statistical tests. *P* < 0.05 was considered significant. Supplementary methods was supplied as individual Additional file 1 [17].

## Results

### RNF43 was associated with E-cadherin downregulation in lung adenocarcinoma in the context of c-Src activation

Hakai is characterized as an E-cadherin-binding protein, and E3 ubiquitin ligase induces the ubiquitination of E-cadherin following the c-Src-mediated tyrosine phosphorylation of E-cadherin in Madin Darby canine kidney (MDCK) epithelial cells [13]. To generalize and test these results in human lung adenocarcinoma, protein extracts from 60 pairs of cancerous and paracancerous tissues were incubated with high-profile microarrays containing monoclonal antibodies against 620 E3 ubiquitin ligases and 30 EMT-related molecules (Additional file 2: Table S1, Additional file 3: Table S2, and Fig. 1a). We investigated the expression of activated c-Src, a prerequisite for E-cadherin ubiquitination and degradation. c-Src was overactivated in lung adenocarcinomas relative to that in paracancerous tissues (Additional file 3: Table S2 and Fig. 1b), and this overactivation was tightly correlated with decreased E-cadherin expression as determined by a protein antibody microarray (Additional file 5: Figure S1A and Fig. 1b). Activated c-Src exclusively phosphorylated Caspase-8 at the tyrosine 380 site (Tyr-380) [18]. Similarly, phosphorylated Caspase-8 was tightly associated with activated c-Src in our study (Additional file 5: Figure S1B and Fig. 1b). Based on the role of E-cadherin depletion in the process of EMT, we explored the relationship between E-cadherin expression and disease progression. In the cohort of patients with resectable lung adenocarcinoma (Additional file 4: Table S3), E-cadherin loss was predictive of worse survival and more aggressive behavior (Additional file 5: Figure S1C and D).

RETRACTED

**Fig. 1:** RNF43 was associated with E-cadherin downregulation in lung adenocarcinoma. **a**, Total protein extracts from cancerous (left) and paracancerous (right) tissues were analyzed by antibodies and processed for high-throughput immunoblotting using protein antibody microarrays consisting of 650 antibodies. **b**, The microarray analysis described in A unveiled the differences in protein expression between cancerous and paracancerous tissues, revealing significant upregulation (red color) of RNF43 and p-Src in lung adenocarcinoma. The green and yellow colors represent equal signals and downregulation (E-cad) in lung adenocarcinoma. **c**, Luciferase-based siRNA library screen for human E3 ligases identified multiple E3 candidates upon knockdown in SUM-E-cad-Luc/R-Luc cells, which increased luciferase activity by more than 4-fold. **d**, Immunohistochemical staining for RNF43 and E-cadherin was performed at high magnification (× 400)

Surprisingly, Hakai, a well-known E3 ligase for E-cadherin, was almost undetectable in 60 lung adenocarcinomas and was not linked to E-cadherin downregulation (Additional file 2: Table S1and Fig. 1a), raising the question of whether Hakai can dampen E-cadherin expression in lung adenocarcinoma via c-Src activation. To elucidate the candidate E-cadherin E3 ligase in lung adenocarcinoma, we utilized previously reported procedures (Additional file 5: Figure S1E) [19]. We knocked down individual human E3 ligases in SUM-E-cadherin-Luc/R-Luc cells using pooled siRNAs (3 siRNAs) and searched for E3 ligase in A549 cells with c-Src activation, which increased the luciferase activity greater than 4-fold. Then, immunoprecipitation was used to confirm the interaction between the candidates and E-cadherin (data not shown). Accordingly, RNF43 markedly affected the SUM-E-cadherin-Luc to R-Luc ratio upon immunoprecipitation with E-cadherin, inducing the highest fold change of 7.6 among all the proteins analyzed (Fig. 1c). In addition, out of 620 E3 ubiquitin ligases, RNF43, a transmembrane E3 ubiquitin ligase, was most ubiquitously detected and most markedly upregulated (by 28-fold) in cancerous tissues compared with that in paired tissues (Additional file 2: Table S1, Fig. 1a and b), which was further confirmed by immunohistochemistry (IHC) analysis (Fig. 1d). Together, these results suggest that RNF43 potentially downregulates E-cadherin in lung adenocarcinoma in the context of c-Src activation.

RETRACTED

### C-Src was overactivated through its interaction with Caspase-8 to promote the metastasis of lung adenocarcinoma cells

Previous reports indicated that Caspase-8 is selectively phosphorylated at Tyr-380 (pY380) by c-Src to block tumor cell apoptosis [18, 20, 21]. In parallel, we observed that the c-Src-Caspase-8 interaction efficiently overactivates c-Src to induce EMT [14]. However, exploring the detailed mechanism underlying c-Src activation was necessary. Initially, c-Src and Caspase-8 expression was evaluated in lung adenocarcinoma-derived cell lines (Additional file 6: Figure S2A), including A549 (Casp8^+^Src^+^) and H522 (Casp8^−^Src^+^) cells. Endogenous Caspase-8 or c-Src was knocked down in A549 cells with the lentiviral delivery of Caspase-8 or c-Src shRNA (Fig. 2a). pY380-Caspase-8 was not detected in the c-Src-knockdown A549 cells (Fig. 2a), while c-Src phosphorylation at Tyr-416 (activated c-Src) was obviously compromised in the Caspase-8-knockdown A549 cells (Fig. 2a). The re-expression of Caspase-8 in H522 cells lacking endogenous Caspase-8 elicited a significant increase in c-Src activity (Fig. 2b). The fluorometric substrate assay showed increased c-Src activity among A549 + control shRNA and H522 + Casp8 WT cells (Fig. 2c). Notably, transfecting the Caspase-8 mutant Y380A Caspase-8 (Casp8 Y380A) into Caspase-8-deficient H522 cells via lentivirus failed to restore c-Src activation like wild-type Caspase-8 (Casp8 WT) (Fig. 2b and c), implying an indispensable role for Tyr-380 in Caspase-8-mediated c-Src activation. The association of pY416-Src with Caspase-8 in A549 cells was confirmed in the complex immunoprecipitated by an anti-Caspase-8 antibody (Fig. 2d), and pY380-Caspase-8 interacted with c-Src in the extracts of A549 cells transfected with control shRNA and H522 cells transfected with Casp8 WT (Fig. 2d). As expected, Y380A Caspase-8 was dissociated with pY416-Src (Fig. 2d). To test whether pY380-Caspase-8 interacted with c-Src via the c-Src SH2 domain, the recombinant SH2 domain of c-Src fused to GST was generated for use in pulldown assays. pY380-Caspase-8 was efficiently pulled down by c-Src SH2-GST (Fig. 2d), and pY380-Caspase-8 enhanced c-Src activation via binding to the SH2 domain of c-Src.

**Fig. 2:** c-Src was activated through c-Src-Caspase-8. **a**, Immunoblotting analysis of phospho-Caspase-8 (pY380-Casp8) and phospho-c-Src (pY416-Src) in A549 + control/Casp8/c-Src shRNA cells plated on fibronectin (10 μg/ml) for the indicated amounts of time. **b**, Immunoblotting analysis of phospho-Caspase-8 and phospho-c-Src in A549 cells transfected with a control vector and H522 cells transfected with adenovirus encoding the control vector, wild-type Caspase-8 (Casp8 WT) or Y380A Caspase-8 (Casp8 Y380A) plated on fibronectin (10 μg/ml) for 1 day. **c**, A549 cells (upper panel) transfected with either control shRNA or Casp8 shRNA via lentivirus were plated on fibronectin (10 μg/ml) in the presence of a c-Src-specific fluorescent substrate, and fluorescence was recorded as a function of time (*t* test, *, *P* < 0.05). H522 cells (lower panel) transfected with a control vector, Casp8 WT, or Casp8 Y380A via adenovirus were plated on fibronectin (10 μg/ml) in the presence of a c-Src-specific fluorescent substrate, and fluorescence was recorded as a function of time (*t* test, *, *P* < 0.05). **d**, pY380-Casp8 and pY416-Src immunoblot analysis of A549 + control shRNA and H522 + control vector/Casp8 WT /Casp8 Y380A cell extracts immunoprecipitated with anti-Casp8 or anti-HA after tumor cells were allowed to attach to fibronectin (10 μg/ml) for 4 days. pY380-Casp8 immunoblot analysis was performed by a pulldown assay with 2 μg of GST-SH2 domains from c-Src and Abl; GST itself was used as a control. Anti-Casp8 and anti-c-Src immunoblotting of immunoprecipitated total cell lysates is shown at the bottom. **e**, Ectopically grown A549 (upper panel)/H522 (lower panel) tumors were surgically removed. Biweekly quantification of bioluminescence showed accelerated tumor growth and increased spontaneous metastasis in the mice implanted with A549 + control shRNA and H522 + Casp8 WT cells (*t* test, * *P* < 0.05). Data are presented as the mean ± SD. **f**, Total cumulative incidences of micrometastasis confirmed by immunostaining in the tumor-implanted mouse cohorts (*χ*^*2*^ test, *, *P* < 0.05). Micrometastatic events in various BALB/c nude mouse organs were confirmed by immunostaining. Tissue sections were scored as positive or negative based on the presence or absence of detectable micrometastasis

We tested the effects of Caspase-8-c-Src on distant spontaneous metastasis after primary tumor removal in nude mice. To ensure equal tumor burdens, resected tumors were weighed at the same sizes. Mice implanted with A549 + control shRNA and H522 + Casp8 WT cells showed significantly increased spontaneous metastatic tumor burdens (Fig. 2e) as measured by bioluminescence (Additional file 6: Figure S2B). HE staining confirmed micrometastasis in the nude mouse organs, and representative staining is shown in Additional file 6: Figure S2C. Significantly increased micrometastatic incidences and extended tumor distributions were detected in the mice inoculated with Casp8^+^Src^+^ A549/H522 cells (Fig. 2f and Additional file 6: Figure S2D and S2E), which corresponded to a shorter OS (Additional file 6: Figure S2F). The Y380A mutation in the Caspase-8 holoprotein obviously attenuated the metastasis of H522 cells (Fig. 2f and Additional file 6: Figure S2D and S2E). Together, these results suggested that Caspase-8-c-Src potently promoted c-Src activation to facilitate tumor cell dissemination from lung adenocarcinoma.

RETRACTED

### RNF43 ubiquitinated and degraded E-cadherin in lung adenocarcinoma cells with c-Src activation

Activated c-Src was reported to phosphorylate E-cadherin at the tyrosine sites to initiate the Hakai-induced ubiquitination and degradation of E-cadherin [12, 13]. With the linkage of RNF43 to decreased E-cadherin expression and ubiquitous c-Src activation in lung adenocarcinoma, we expected to elucidate the mechanism by which RNF43 interacts with E-cadherin in the context of c-Src activation. RNF43 was frequently associated with Hakai deficiency in lung adenocarcinoma cell lines (Fig. 3a), while E-cadherin was obviously upregulated upon c-Src inactivation (Fig. 3a). Caspase-8-expressing A549 and H522 cells displayed c-Src hyperactivity with decreased E-cadherin (Fig. 3b and c). The Caspase-8-induced activation of c-Src ignited the ubiquitination of E-cadherin in RNF43-expressing A549 and H522 cells, which was impaired by RNF43 knockdown via an shRNA targeting RNF43 (Fig. 3d), suggesting that RNF43 might induce the ubiquitination and degradation of E-cadherin following c-Src activation. Using an antibody against E-cadherin, RNF43 was markedly coimmunoprecipitated with E-cadherin (Fig. 3d). Immunofluorescence analysis confirmed the colocalization of E-cadherin with RNF43 on the A549 cell membrane (Fig. 3e), supporting the interaction between E-cadherin and RNF43. Then, the posttranscriptional downregulation of E-cadherin was confirmed by the observance of equal E-cadherin mRNA expression in A549 and H522 cells (Fig. 3f). To dissect the relationship between E-cadherin ubiquitination and c-Src activation, we overexpressed RNF43 in A549 cells with or without c-Src knockdown. c-Src knockdown hampered E-cadherin ubiquitination (Additional file 7: Figure S3A), while RNF43 overexpression had no impact on E-cadherin ubiquitination in A549 cells with or without c-Src knockdown (Additional file 7: Figure S3A). To confirm the ability of RNF43 to directly ubiquitinate E-cadherin, we isolated RNF43-containing complexes from A549 cells overexpressing RNF43 by immunoprecipitation and examined the ubiquitination activity toward in vitro-translated E-cadherin. A constitutively active c-Src, Src Y527F, was added to the in vitro reaction system. In the presence of recombinant ubiquitin plus the E1 and E2 enzymes, the RNF43 complex promoted E-cadherin ubiquitination in a manner dependent on c-Src activation (Additional file 7: Figure S3B).

RETRACTED

**Fig. 3:** Activated c-Src mediated the ubiquitination and degradation of E-cadherin in lung adenocarcinoma cells. **a**, Immunoblot analysis of c-Src, pY416-Src (p-Src), E-cadherin (E-cad), RNF43, Hakai and β-actin in the human lung adenocarcinoma cell lines A549, NCI-H522, NCI-H1975, NCI-H1623 and NCI-H2073. **b**, A549 cells were stably transfected with lentivirus containing control or Caspase-8 shRNA (Cap8 KD). Caspase-8, p-Src, c-Src, E-cad and β-actin in total cell lysates (TCLs) were detected by western blot. **c**, Caspase-8-deficient H522 cells were stably transfected with a control vector or wild-type Caspase-8 via adenovirus. Caspase-8, p-Src, c-Src, E-cad and β-actin in TCLs were detected by western blot. **d**, The TCLs of A549 and H522 cells in which c-Src was activated were subjected to immunoprecipitation (IP) using an anti-E-cadherin antibody. Ubiquitinated (Ubi-) E-cadherin was detected by western blot (*upper blot*). The blot was then stripped and reprobed for RNF43 (*second from upper panel*). RNF43, E-cadherin and β-actin were in TCLs detected by western blot (*lower blot*). **e**, A549 cells were allowed to attach to dishes for 12 h and then assessed by confocal microscopy using antibodies against E-cadherin and RNF43. Scale bars, 10 μm. **f**, E-cadherin mRNA was examined in A549 + control/Caspase-8 shRNA cells (Casp8 KD) and in H522 + control vector/wild-type Caspase-8 cells

We next asked whether E-cadherin was degraded through proteasome-mediated proteolysis on the basis of its ubiquitination. MG132, a cell-permeable proteasome inhibitor, efficiently eluded E-cadherin degradation in A549 and H522 cells (Additional file 7: Figure S3C). To identify the E-cadherin ubiquitination site, we individually mutated three lysines in its cytoplasmic domain, including K816A, K855A, and K871A, of which E-cad K816A failed to restore E-cadherin ubiquitination (Additional file 7: Figure S3D), indicating that RNF43 ubiquitinated E-cadherin at the cytoplasmic lysine 816. The destination of ubiquitinated proteins is determined by the ubiquitin attachment and type of polyubiquitin chain. When ubiquitin was tagged with intracellular substrates via lysine 48/63 (K48/63)-linked polyubiquitin chains, proteins were subjected to 26S proteasome-mediated recognition and proteolysis [22–24]. Using MS/MS analysis and database searching, we found that only the K48 polyubiquitin chain was added (Additional file 7: Figure S3E, *left*), which was confirmed by the immunoprecipitation of endogenous E-cadherin followed by immunoblotting with a K48 or K63 polyubiquitin chain-specific antibody (Additional file 7: Figure S3E, *right*). Taken together, these results indicate that RNF43 degrades E-cadherin through its ubiquitination at the K816 site in the context of c-Src activation in lung adenocarcinoma.

RETRACTED

### RNF43-induced E-cadherin degradation initiates the EMT phenotype via allowing the translocation of β-catenin into the nucleus

The metastasis of cancer cells from primary tumors is thought to occur by the process of EMT [8, 25]. E-cadherin loss was characterized as an initiator of EMT in cancer cells [26–28]. We next wanted to investigate whether RNF43-induced E-cadherin degradation was responsible for the EMT promotion of lung adenocarcinoma metastasis. Over the course of 5 days, A549 cells transfected with a lentiviral shRNA targeting RNF43 (RNF43 KD) presented no EMT morphological characteristics compared with A549 cells transfected with control shRNA (Fig. 4a). We subsequently explored the role of RNF43 in spontaneous distant metastasis after primary tumors weighing the same size were removed from nude mice. Mice implanted with A549 + control shRNA cells had a significantly increased tumor burden, and metastasis occurred in all ten mice in the group (Fig. 4b) as measured by bioluminescence (Fig. 4c). As determined by HE staining (Fig. 4d), markedly increased metastatic incidences and extended tumor distributions were observed in mice inoculated with A549 + control shRNA cells (Fig. 4e), which corresponded with a worse OS (Fig. 4f).

**Fig. 4:** RNF43 enhanced lung adenocarcinoma cell metastasis through EMT. **a**, Phase contrast microscopy of A549 + control shRNA cells (Control) or RNF43 shRNA cells (RNF43 KD) plated on dishes over a 5-day period. Scale bars, 50 μm. **b**, Ectopically grown A549 cells were surgically removed. Biweekly quantification of bioluminescence showed accelerated tumor growth and increased spontaneous metastasis in the mice implanted with A549 + Control cells relative to that in mice implanted with A549 + RNF43 KD cells (*t* test, *, *P* < 0.05). Data are presented as the mean ± SD. **c**, Representative bioluminescence images of tumor cells before and after primary tumor resection (10 and 30 days after resection). **d**, HE staining of micrometastasis to bone, lung, liver, and brain tissue. Scale bars, 100 mm. **e**, Total cumulative incidences of micrometastasis in the tumor-implanted mouse cohorts as confirmed by immunostaining (*χ*^*2*^ test, *, *P* < 0.05). Micrometastatic events in various BALB/c nude mouse organs were confirmed by immunostaining. Tissue sections were scored as positive or negative based on the presence or absence of detectable micrometastasis. **f**, Kaplan-Meier survival analysis of the corresponding mice showed significantly shorter survival times for mice implanted with A549 + Control cells compared with that of mice implanted with A549 + RNF43 KD cells (log-rank test, **, *P* < 0.01)

A549 + control shRNA cells exhibited EMT molecular features with decreased E-cadherin expression and increased Vimentin expression (Fig. 5a). Although Slug, Snail, Twist, Fibronectin, and N-cadherin were proposed to affect EMT [29–31], their levels were not markedly different in A549 cells transfected with control, RNF43, or c-Src shRNAs via lentivirus (Fig. 5a). Immunoprecipitated E-cadherin conjugated with ubiquitin was pronounced in the RNF43-expressing A549 cells (Fig. 5b), and translocation of β-catenin into the nucleus was markedly increased (Fig. 5b). Although GSK-3β was reported to regulate the distribution and degradation of β-catenin via phosphorylating β-catenin at Ser33, Ser37 and Thr41 [32], GSK-3β and phospho-β-catenin (p-β-catenin) were comparably expressed in various A549 cells (Fig. 5b). Coimmunoprecipitation with an antibody specific for β-catenin revealed that the interaction between GSK-3β and β-catenin was not affected by the silencing of RNF43 or c-Src (Fig. 5c), whereas E-cadherin was not involved in the immunocomplex of A549 cells with control shRNA (Fig. 5c). Thus, E-cadherin degradation more likely promoted the release of cytoplasmic β-catenin into the nucleus. Nuclear β-catenin acts as a transcription factor to affect a wide range of genes by forming a transcriptional complex with TCF-4 [33, 34], and we observed that β-catenin interacted with TCF-4 in A549 cells (Fig. 5c). We next explored whether β-catenin translocated into the nucleus functioned in the transcription factor complex to govern the mRNA levels of E-cadherin and Vimentin. An antibody against β-catenin, 7A7, was delivered to prevent its nuclear translocation into A549 cells, and the sequestration of β-catenin in the cytoplasm vastly diminished the protein and mRNA levels of Vimentin (Fig. 5d and e). The delivery of 7A7 and knockdown of TCF-4 had no effects on E-cadherin mRNA expression (Fig. 5e). RNF43 was determined to be a direct target of the TCF-4/β-catenin complex because RNF43 transcription was inhibited in A549 cells treated with 7A7 and TCF-4 knockdown (Fig. 5d and e). As expected, Wnt-responsive element (WRE) was detected in the promoter regions of Vimentin and RNF43. ChIP assays using antibodies against TCF-4 and β-catenin showed that the promoter regions of Vimentin and RNF43 were bound to the TCF-4/β-catenin complex (Fig. 5f and g). Furthermore, we constructed a reporter gene (luciferase) assay system with the promoter variants, as shown in Fig. 5h, which were transiently transfected into A549 cells. The reporter activities of cells expressing the Vimentin and RNF43 promoters were significantly increased, and this activity was impaired by deleting WRE from the promoter regions (Fig. 5i). The luciferase activity was not changed in A549 cells transfected with E-cadherin promoter-luciferase (Fig. 5i). Our data suggested that RNF43-induced E-cadherin degradation followed by c-Src activation initiated the EMT phenotype via allowing the translocation of β-catenin into the nucleus. To test whether the loss of E-cadherin was sufficient to maintain the EMT phenotype, we knocked down E-cadherin in H522 cells via the lentiviral delivery of E-cadherin shRNA, and E-cadherin knockdown was sufficient to trigger both EMT along and the nuclear translocation of β-catenin (Additional file 8: Figure S4A and B).

RETRACTED

**Fig. 5:** RNF43-induced E-cadherin ubiquitination and degradation initiated EMT phenotype via allowing β-catenin to translocate into the nucleus in a c-Src-dependent manner. **a**, A549 cells were stably transfected with the lentiviral control shRNA, RNF43 shRNA, or c-Src shRNA. Snail, Slug, Twist, E-cadherin (E-cad), Vimentin, Fibronectin, N-cadherin (N-cad), and β-actin in total cell lysates (TCLs) were detected by western blot. **b**, A549 cells stably transfected with lentiviral control shRNA, RNF43 shRNA, or c-Src shRNA were seeded overnight. TCLs were subjected to immunoprecipitation (IP) using an anti-E-cadherin antibody. Ubiquitinated E-cadherin was detected by western blot with an anti-ubiquitin antibody (*upper blot*). Phospho-β-catenin (p-β-catenin), β-catenin, GSK-3β, RNF43, and β-actin in TCLs were detected by western blot (*middle blot*). β-catenin was detected in the nuclear extract of A549 cells (*lower blot*). **c**, The TCLs of A549 cells stably transfected with lentiviral control shRNA, RNF43 shRNA, or c-Src shRNA were subjected to IP using an anti-β-catenin antibody. E-cadherin, GSK-3β, TCF-4, and β-catenin were detected by western blot. **d**, A549 cells were treated with an shRNA either not targeting TCF-4 (Control) or targeting TCF-4 (TCF-4). The in vitro β-catenin antibody 7A7 was delivered into A549 cells. Immunoblot analysis of LaminA/C (loading control), TCF-4, E-cad, Vimentin, and nuclear/total β-catenin was performed using appropriate antibodies. **e**, A549 cells were treated with an shRNA either not targeting (Control) or targeting TCF-4 (TCF-4). The in vitro β-catenin antibody 7A7 was delivered into A549 cells. The mRNA levels of E-cad, Vimentin, and RNF43 were examined by RT-PCR. GAPDH mRNA was used to confirm equal loading. **f** and **g**, β-catenin and TCF-4 chromatin immunoprecipitation (ChIP) in A549 cells. PCR was carried out using primers specific for the promoter regions of E-cad, Vimentin, and RNF43. One-fifth of the input DNA from each sample was also amplified and designated as Input. **h**, Schematic representation of reporter plasmids containing the control vector, E-cadherin promoter, Vimentin promoter, Vimentin promoter with WRE deletion (Vim mut), RNF43 promoter, and RNF43 promoter with WRE deletion (RNF43 mut). **i**, A549 cells were transiently transfected with the reporter plasmids described in **f**. Luciferase activities were measured in triplicate (mean ± SD, *t* test, *, *P* < 0.05)

RETRACTED

### C-Src was responsible for RNF43-mediated E-cadherin ubiquitination through E-cadherin phosphorylation at tyrosine 797

To profoundly dissect the relationship between c-Src activation and E-cadherin degradation, we constructed HA-tagged variants of c-Src, including wild-type c-Src (control, Src WT) and constitutively active c-Src with the point mutation of Y527F (Src Y527F) in p-Src-null H522 cells. Exogenous Src Y527F significantly elevated c-Src activity, leading to E-cadherin ubiquitination and degradation (Fig. 6a and b). Activated c-Src was coimmunoprecipitated with E-cadherin, and an E-cadherin phosphotyrosine was detected in the immunoprecipitated complex using a nonspecific phosphotyrosine antibody (Fig. 6b). Then, we investigated whether activated c-Src was sufficient to attain the EMT phenotype in H522 cells. Compared with that achieved with Src WT, constitutively active c-Src promoted EMT morphological changes and metastasis of H522 cells (Fig. 6c). MALDI-mass spectrometry was applied to identify the phosphotyrosine site of E-cadherin. Purified E-cadherin was cleaved by CNBr, and the MS spectrum revealed an m/z peak at 1599.58 Da, corresponding to an 80 Da shift of the m/z cleavage fragment at 1519.60 Da (Fig. 6d). The CNBr cleavage peptide, in which tyrosine 797 is phosphorylated and conserved across diverse species, was recovered from the MALDI spectrum (Fig. 6d). However, three closely spaced tyrosines, tyrosine 755–757, in the cadherin homology 2 (CH2) domain were previously demonstrated to mediate E-cadherin phosphorylation in a modified yeast 2-hybrid system [13]. As a result, HA-tagged Y755-757F, Y797F and wild-type E-cadherin (E-cad WT) were constructed and transfected into E-cadherin-knockdown A549 cells. The phosphorylation and ubiquitination of Y755-757F E-cadherin induced the EMT phenotype in A549 cells, like E-cad WT (Fig. 6e, f, and g), whereas Y797F E-cadherin impaired the phosphorylation of E-cadherin and failed to restore tumor cell aggressiveness via sequestering β-catenin, leading to abolished changes in EMT biomarkers and morphology (Fig. 6e, f, and g). Together, these results suggest that E-cadherin phosphorylated at tyrosine 797 by activated c-Src initiated E-cadherin ubiquitination and degradation, thus facilitating the EMT phenotype in lung adenocarcinoma.

RETRACTED

**Fig. 6:** c-Src underlay RNF43-mediated E-cadherin ubiquitination through E-cadherin phosphorylation at tyrosine 797. **a**, H522 cells were stably transfected with wild-type c-Src (Src WT) and a constitutively active c-Src, Src Y527F. p-Src, c-Src, E-cadherin (E-cad), Vimentin, RNF43, total β-catenin, and β-actin via adenovirus and detected by western blot analysis of total cell lysates (TCLs) (*Upper blot*). β-catenin in the nuclear extract was evaluated using an antibody against β-catenin (*lower blot*). **b**, TCLs were subjected to immunoprecipitation (IP) using an anti-E-cadherin antibody. Ubiquitinated E-cadherin was detected with an anti-ubiquitin antibody. p-Src, RNF43, nonspecific phosphorylated tyrosine of E-cadherin (p-Tyr-100), and E-cadherin in the immunocomplex were detected by western blot. **c**, EMT morphological changes and metastatic incidences in H522 cells transfected with Src WT and Src Y527F (*χ*^*2*^ test, *, *P* < 0.05). Scale bars, 50 μm. **d**, Tyrosine 797 of E-cadherin was conserved across various species (*upper panel*). MALDI-mass spectrometry analysis of CNBr-cleaved endogenous E-cadherin expression in A549 cells with or without endogenous c-Src (*lower panel*). **e**, E-cadherin-knockdown A549 cells transfected with unmutated E-cadherin (E-cad WT) or E-cadherin mutated at Y755-757F (E-cad Y755-757F) or Y797F (E-cad Y797F) were lysed to obtain TCLs. E-cadherin (anti-HA) was immunoprecipitated from TCLs and probed for ubiquitin-E-cadherin, p-Src, nonspecific phosphorylated tyrosine of E-cadherin, RNF43, and E-cadherin (anti-HA) by western blot. **f**, E-cadherin-knockdown A549 cells transfected with HA-tagged E-cad WT, E-cad Y755-757F, or E-cad Y797F were lysed to obtain TCLs. p-Src, c-Src, Vimentin, E-cadherin (anti-HA), RNF43, total β-catenin, and β-actin were detected by western blot analysis of the TCLs (*upper blot*). Nuclear extracts were subjected to western blot analysis of β-catenin (*lower blot*). **g**, EMT morphological changes and metastatic incidences in E-cadherin-knockdown cells transfected with HA-tagged E-cad WT, E-cad Y755-757F, or E-cad Y797F (*χ*^*2*^ test, *, *P* < 0.05). Scale bars, 50 μm

RETRACTED

### Frz8 was required for the RNF43-induced ubiquitination and degradation of E-cadherin

Wnt signaling induced numerous cellular responses, including EMT [35]. Ten Frz proteins have been identified in mammals as Wnt protein receptors and initiate Wnt signaling, while RNF43 has been demonstrated to ubiquitinate the ectodomain of Frz, leading to its inversion and degradation in a Dishevelled (Dvl)-dependent manner [36–38]. Previous studies indicated that the CRD of Frz and the PA of RNF43 are needed for the interaction between Frz and RNF43 [39], which raises the question of how RNF43 ubiquitinates phosphorylated E-cadherin despite not having a CRD. It was hypothesized that the Frz protein might trigger the active conformation of RNF43 to initiate E-cadherin ubiquitination. We initially observed that RNF43 prohibited Frz8 ubiquitination and degradation in Dvl3-deficient A549 and H522 cells (Fig. 7a and b). Notably, Frz8 knockdown in A549 cells impaired E-cadherin downregulation by protecting E-cadherin from RNF43-mediated ubiquitination (Fig. 7c). This result suggests that Frz8 is critical for the initiation of E-cadherin ubiquitination and degradation. Moreover, we constructed and transfected a variety of RNF43 and Frz8 mutants into RNF43-knockdown/Frz8-knockdown A549 cells (Fig. 7d and Additional file 9: Figure S5A), revealing that the CRD of Frz8 interacted with the PA of RNF43 to facilitate E-cadherin ubiquitination and degradation (Fig. 7e and Additional file 9: Figure S5B). Feng Cong and coworkers reported that Dvl is a dual function adaptor that functions to recruit negative regulators, such as RNF43, to Wnt receptors and thus ensure proper control of pathway activity [38]. We postulated that Dvl3 deficiency might act as a key effector to facilitate RNF43-mediated E-cadherin ubiquitination and impair RNF43-mediated Frz8 ubiquitination. The re-expression of Dvl3 potently impeded the ubiquitination and degradation of E-cadherin by prohibiting the RNF43-E-cadherin interaction (Additional file 9: Figure S5C), while Dvl3 in A549 cells restored the ubiquitination and degradation of Frz8 through the recruitment of RNF43 (Additional file 9: Figure S5D). Thus, Dvl3 was thought to promote the ubiquitination of E-cadherin by RNF43 based on Frz8.

**Fig. 7:** Frz8 was required for the RNF43-induced ubiquitination of phosphorylated E-cadherin. **a**, Immunoblot analysis of Frz8, Frz2, Dishevelled 3 (Dvl3), LGR6, and β-actin in A549 and H522 cells. **b**, A549 and H522 cells stably transfected with control shRNA or RNF43 shRNA (RNF43 KD) via adenovirus were seeded overnight. The total cell lysates (TCLs) were subjected to immunoprecipitation (IP) using an anti-Frz8 antibody. Ubiquitinated Frz8 was detected by western blot with an anti-ubiquitin antibody (*upper blot*). Frz8 and RNF43 in the TCLs were detected by western blot (*lower blot*). **c**, A549 cells stably transfected with control shRNA or Frz8 shRNA (Frz8 KD) via lentivirus were seeded overnight. The TCLs were subjected to IP using an anti-E-cadherin antibody. Ubiquitinated E-cadherin was detected by western blot with an anti-ubiquitin antibody (*upper blot*). E-cadherin, Frz8, and β-actin in the TCLs were detected by western blot (*lower blot*). **d**, Schematic representation of reporter plasmids containing full-length RNF43 and two truncated versions of RNF43 as shown. **e**, RNF43-knockdown A549 cells stably transfected with RNF43, RNF43-R, or RNF43-P via adenovirus were seeded overnight. The TCLs were subjected to IP using anti-E-cadherin and anti-HA antibodies. Ubiquitinated E-cadherin, E-cadherin, Frz8, and HA were detected by western blot (*upper and middle blot*). E-cadherin and β-actin in the TCLs were detected by western blot (*lower blot*). **f**, A549 cells treated with DMSO (Control) or monoclonal antibodies (10.0 mmol/L) against the cysteine-rich domain (CRD) of Frz8 and the RNF43 protease domain (PA) were seeded overnight. The TCLs were subjected to IP using an anti-E-cadherin antibody. Ubiquitinated E-cadherin, RNF43, and E-cadherin were detected by western blot (*upper blot*). E-cadherin, Vimentin, and β-actin in the TCLs were detected by western blot (*middle blot*). β-catenin was detected in the nuclear extract (*lower blot*). **g**, A549 cells treated with DMSO (Control) or monoclonal antibodies (10.0 mmol/L) against the cysteine-rich domain (CRD) of Frz8 and the RNF43 protease domain (PA) were seeded overnight. The TCLs were subjected to IP using an anti-RNF43 antibody. Frz8, RNF43, and E-cadherin were detected by western blot. **h**, EMT morphological changes and metastatic incidences in A549 cells treated with DMSO (Control) or monoclonal antibodies (10.0 mmol/L) against the cysteine-rich domain (CRD) of Frz8 and the RNF43 protease domain (PA) (*χ*^*2*^ test, *, *P* < 0.05). Scale bars, 50 μm. **i**, A549 cells treated with DMSO (Control) and RSOP1–4 were seeded overnight. The TCLs were subjected to IP using anti-E-cadherin and anti-Frz8 antibodies. Ubiquitinated E-cadherin and RNF43 were detected by western blot (*upper and middle blot*). E-cadherin and β-actin in the TCLs were detected by western blot (*lower blot*)

We investigated whether monoclonal antibodies against the CRD of Frz8 and the PA of RNF43 affected the fate of tumor cells. Intriguingly, a monoclonal antibody specific for the CRD of Frz8 efficiently inhibited EMT changes and aggressive behavior by blocking the interaction between Frz8 and RNF43 (Fig. 7f and g). A monoclonal antibody specific for the PA of RNF43 did not exert the same antimetastatic effect as that specific for the CRD of Frz8 (Fig. 7f and g), partially because the binding of RNF43 to E-cadherin was not completely blocked (Fig. 7h). R-spondin (RSPO) was proven to naturally intercept RNF43-Frz and thus rescue Frz degradation by interacting with the leucine-rich repeat-containing G protein-coupled receptor (LGR), which is expressed in A549 and H522 cells (Fig. 7a) [37, 40]. RSPO had no effects on the interplay between Frz8 and RNF43 and failed to restore E-cadherin expression in A549 cells (Fig. 7i). In summary, Frz8 was required to trigger the RNF43-induced ubiquitination of phosphorylated E-cadherin in lung adenocarcinoma cells deficient of Dvl3.

RETRACTED

As RNF43 and ZNRF3 are homologous molecules, their amino acid sequences are 30% identical [41]. Interestingly, ZNRF3 expression in lung adenocarcinoma tissues was rare compared with that of RNF43 (Additional file 2: Table S1). The re-expression of ZNRF3 allowed E-cadherin ubiquitination and was thus responsible for the EMT and metastasis of RNF43-knockdown A549 cells (Additional file 9: Figure S5E and F).

## Discussion

Genomic development has provided opportunities for the integrative analysis of gene expression using serial analysis of gene expression and cDNA microarray [42, 43]. However, the mRNA expression level does not always accurately reflect the level of the corresponding protein or identify changes in the posttranscriptional modification of proteins. Therefore, the analysis of differences in proteins is important to complement studies. A protein antibody microarray containing monoclonal antibodies against human 620 E3 ubiquitin ligases and 30 Wnt signaling molecules was generated in the search for brand-new targets of E3 ubiquitin ligases in lung adenocarcinoma. Fujita and coworkers showed that Hakai functions as an E3 ubiquitin ligase to ubiquitinate and degrade phosphorylated E-cadherin by c-Src [12, 13]. Our data revealed that Hakai was undetectable in lung adenocarcinoma, while E-cadherin was significantly downregulated, accompanied by c-Src activation, raising the question of whether any potential E3 ubiquitin ligases target E-cadherin. Out of 620 E3 ubiquitin ligases, RNF43 expression was remarkably upregulated in lung adenocarcinomas compared with that in noncancerous tissues. RNF43 belongs to a small set of proteins that bear the hallmark sequences of a ubiquitin ligase and a transmembrane region, identified in the earliest discovery of the adult stem cell surface [44]. Bon-Kyoung Koo and coworkers showed that RNF43 reduced Wnt signals by selectively ubiquitinating Frz receptors, thereby targeting Wnt receptors for degradation as an antitumor factor [36, 41]. Our study elucidated a novel role of RNF43 as a key proinvasive factor to directly ubiquitinate E-cadherin at Lys-816, targeting its degradation and thus potentiating lung adenocarcinoma metastasis through inducible EMT. Although ubiquitination is one of the most common mechanisms of targeting membrane proteins for their degradation by proteasomes, many membrane proteins have distinct fates [12]. The roles of different linkages in polyubiquitins have been elucidated in recent years. Linkage via Lys-48 is mainly used for targeting the proteasome, and that via Lys-63 appears to play an important role in DNA damage tolerance, inflammatory responses, and ribosomal protein synthesis [22]. The present study revealed that RNF43 ubiquitinated E-cadherin through the Lys-48 linkage, leading to its eventual degradation. ZNRF3 and RNF43 exhibit amino-terminal extracellular regions of uncharacterized topology, and the sequences of the two proteins are moderately conserved at 39% identity [37]. Compared with RNF43, ZNRF3 was infrequently expressed in lung adenocarcinoma, although ZNRF3 was sufficient to ubiquitinate E-cadherin. Therefore, the alternative expression patterns of RNF43 and ZNRF3 in lung adenocarcinoma will be our interest and focus in future studies.

RETRACTED

EMT is a dynamic process that leads to cellular aggressiveness with decreased adhesion, and its transdifferentiation is characterized by decreased epithelial markers and increased mesenchymal markers [45]. E-cadherin downregulation abolished the E-cadherin-mediated sequestering of β-catenin, allowing its translocation into the nucleus to regulate the expression of a wide range of genes, including Vimentin [46]. β-catenin translocated in the nucleus partners with DNA-binding proteins, such as TCF-4, that recognize specific sequence motifs in the promoters and enhancers of target genes [33, 47]. We showed that the RNF43-induced degradation of E-cadherin was essential for triggering EMT through the nuclear translocation of β-catenin in lung adenocarcinoma cells. The fact that the nuclear translocation of β-catenin increased Vimentin transcription was supported by our findings that treatment with a β-catenin antibody suppressed Vimentin mRNA expression via impairing β-catenin nuclear translocation, and TCF-4 knockdown diminished Vimentin mRNA expression. Interestingly, the protein and mRNA levels of E-cadherin were not altered by treatment with the β-catenin antibody or TCF-4 knockdown, indicating the posttranscriptional downregulation of E-cadherin. In addition, RNF43 mRNA expression was upregulated by the binding of a β-catenin/TCF-4 transcriptional complex to the WRE element in the promoter region of RNF43. Therefore, RNF43 was characterized as a β-catenin target gene that underlies a positive cycle from E-cadherin downregulation to RNF43 upregulation. Moreover, our data revealed that E-cadherin loss was sufficient to induce and maintain EMT in lung adenocarcinoma.

c-Src-mediated E-cadherin phosphorylation was shown to be required for its ubiquitination and degradation by binding to Hakai, an E3 ubiquitin ligase containing the SH2, RING, zinc-finger and proline-rich domains [13]. c-Src is conventionally involved in tumorigenesis and metastatic cascades [48]. To date, striking and increasing evidence supports the nonapoptotic roles of Caspase-8 [49]. A linkage between Caspase-8 and c-Src was confirmed by observation that cell stimulations with metastasis-promoting factors led to c-Src-mediated Caspase-8 phosphorylation on Tyr-380. We found that the phospho-Tyr-380 of Caspase-8 reversely enhanced c-Src activation via docking to the SH2 domain of c-Src, suggesting that the interaction between Caspase-8 and c-Src results in c-Src hyperactivity, a prerequisite for the RNF43-mediated ubiquitination of E-cadherin. We believe that Caspase-8 phosphorylation via activated c-Src overactivates c-Src, in turn inducing EMT in lung adenocarcinoma. The spontaneous induction of EMT is possible on the basis of the c-Src-Caspase-8 interaction. As Src family members do not have the ability to autoactivate themselves [48], c-Src was likely activated to some extent, enabling Caspase-8 phosphorylation.

RETRACTED

In our study, constitutively active c-Src in p-Src-null H522 cells strongly promoted the RNF43-mediated E-cadherin degradation, thus releasing β-catenin into the nucleus and mediating EMT via formation of the β-catenin/TCF-4 transcriptional complex. With the abovementioned outcomes, c-Src activation requires much more attention. Tyr-755, Tyr-756 and Tyr-757 in the CH2 domain of E-cadherin mediate E-cadherin phosphorylation in a Hakai-dependent manner [13]. Our results demonstrated that RNF43 mediated the ubiquitination and degradation of phosphorylated E-cadherin by c-Src at Tyr-797. Given previous evidence of a phosphorylated tyrosine site shifting upon c-Src kinase activity, this result raises the possibility that E-cadherin is subjected to Tyr-797 phosphorylation following c-Src activation in lung adenocarcinoma cells through an alternative molecular pathway. More likely, however, the phosphorylation of E-cadherin by c-Src alters the structure of E-cadherin such that it has a higher affinity for the RNF43 RING domain, allowing its ubiquitination. We showed a positive feedback loop among Caspase-8-c-Src-RNF43-E-cadherin-β-catenin-RNF43. Interestingly, cytoplasmic signaling loop programs with cancerous traits occur frequently, which is supported by recent reports on the EMT positive feedback loop [50, 51].

RNF43 has no specific domain for recognizing protein phosphotyrosine sites, and very little information is available to support these novel outcomes. Tadasuke Tsukiyama and coworkers found that suppression of Wnt/β-catenin signaling required interaction between the PA of RNF43 and the CRD of Frz [39], .but whether Frz contribute to RNF43-induced E-cadherin ubiquitination remained in question. Our results revealed that both domains are required for RNF43-induced E-cadherin ubiquitination and that Frz8 triggers RNF43-induced E-cadherin ubiquitination. Surprisingly, Frz8 ubiquitination was not detected in lung adenocarcinoma. Recently, an unexpected role of Dvl3 in promoting Wnt receptor degradation was disclosed [38]. Consistently, Dvl3 balances the E-cadherin and Frz8 degradation induced by RNF43. Frz8-RNF43 without Dvl3 potently triggered RNF43-induced E-cadherin degradation, while Frz8-RNF43-Dvl3 efficiently induced Frz8 ubiquitination. This result indicated that Frz8-RNF43 without Dvl3 might change the conformation of RNF43, particularly in its RING domain, thus leading to the ubiquitination of phosphorylated E-cadherin. Thus, monoclonal antibodies specific for the CRD of Frz8 and the PA of RNF43 were produced to expatiate the likelihood of identifying a novel target for the treatment of lung adenocarcinoma. The Frz8 antibody exerted a more substantial antimetastatic effect than the RNF43 antibody, leading to the speculation that the monoclonal RNF43 antibody was incapable of dissociating RNF43 from phosphorylated E-cadherin. Therefore, the monoclonal antibody against the Frz8 CRD potentially represents a new therapeutic strategy for lung adenocarcinoma.

## Conclusions

Protein antibody microarray analysis and E3 ligase profiling revealed that RNF43 is linked to E-cadherin downregulation in the context of c-Src activation in lung adenocarcinoma tissues. c-Src activated via interaction with Caspase-8 phosphorylates E-cadherin at Tyr-797, triggering RNF43-mediated E-cadherin ubiquitination at the Lys-816 site. This event is responsible for E-cadherin degradation, thus allowing the translocation of β-catenin into the nucleus and upregulation of Vimentin and RNF43 expression. Decreased E-cadherin expression and increased Vimentin expression induces the EMT phenotype and thus enhances tumor cell aggression. Through the ubiquitination and degradation of E-cadherin, RNF43 participates in the regulation of EMT during lung adenocarcinoma metastasis. Moreover, Frz8-RNF43 initiates the ubiquitination of phosphorylated E-cadherin, which can obviously be blocked by a monoclonal antibody against the CRD of Frz8 (Additional file 10: Figure S6).

RETRACTED

## Additional files

Additional file 1: Supplementary methods (DOC 74 kb)

Additional file 2: **Table S1**. List of the human E3s. (PDF 225 kb)

Additional file 3: **Table S2**. List of EMT-related proteins. (PDF 63 kb)

Additional file 4: **Table S3**. Information on E-cad-positive and E-cad-negative patients. (PDF 44 kb)

Additional file 5: **Figure S1.** E-cadherin was predictive of worse survival in patients with lung adenocarcinoma. A, Relationship between E-cadherin and p-Casp8/p-Src. B, Relationship between p-Casp8 and p-Src. C, Kaplan-Meier progression-free survival curves of lung adenocarcinoma patients with negative or positive E-cadherin expression (log-rank test, *P* < 0.001). D, Kaplan-Meier overall survival curves of lung adenocarcinoma patients with negative or positive E-cadherin expression (log-rank test, *P* < 0.05); E, Experimental procedure flow chart for identifying E3 ubiquitin ligase(s) targeting the E-cadherin protein. (JPG 456 kb)

Additional file 6: **Figure S2.** c-Src activation promoted lung adenocarcinoma metastasis. A, Immunoblot analysis of c-Src, p-Src, Caspase-8, p-Casp8 and β-actin in the human lung adenocarcinoma cell lines A549, NCI-H522, NCI-H1975, NCI-H1623 and NCI-H2073. B, Representative bioluminescence images of tumor cells before and after primary tumor resection (days 5 and 30 after resection). C, HE staining of micrometastasis to the lung (upper) and vertebrae of the spinal column (lower). Scale bars, 100 mm. D and E, Total cumulative incidence of micrometastasis in the tumor-implanted mouse cohorts as confirmed by immunostaining (*χ*^*2*^ test, * *P* < 0.05). F, Kaplan-Meier survival curves of the corresponding mice showed significantly decreased survival of the mice cohort implanted with A549 + control shRNA cells compared with that of mice implanted with A549 + Casp8/c-Src shRNA cells (log-rank test, ** *P* < 0.01). (JPG 2077 kb)

Additional file 7: **Figure S3.** RNF43 ubiquitinated E-cadherin**.** A, The TCLs of A549 cells transfected with control shRNA/c-Src shRNA were subjected to IP using an anti-E-cadherin antibody. Ubiquitinated (Ubi-) E-cadherin was detected by western blot (*upper blot*). c-Src, RNF43, and β-actin were detected by western blot analysis of the TCLs (*lower blot*). B, In vitro-translated T7-tagged E-cadherin and a His-tagged active c-Src, Src Y527F, were incubated with immunoprecipitated RNF43 complexes or control IgG in a ubiquitination reaction mixture for 1 h at 30 °C. The reaction was analyzed by T7 immunoblotting. C, Caspase-8-expressing A549 and H522 cells were seeded overnight in the presence or absence of the proteasomal inhibitor MG132 at 25 μg/ml for 3 h. TCLs were subjected to IP using an anti-E-cadherin antibody. E-cadherin and β-actin in TCLs were detected by western blot. D, The TCLs of A549 cells transfected with the E-cad WT, E-cad K816A, E-cad K855A, and E-cad K871A via adenovirus were subjected to IP using an anti-E-cadherin antibody. Ubiquitinated (Ubi-) E-cadherin was detected by western blot (*upper blot*). The blot was then stripped and reprobed for phospho-E-cadherin and E-cadherin. E-cadherin and β-actin were detected by western blot analysis of the TCLs. E, Single-ion chromatographic trace (*left upper*) and full mass spectrum (*left lower*) of isotopically labeled peptides revealed K48 and K63 polyubiquitin chain linkages. A549 cells were seeded overnight. TCLs were subjected to IP using an anti-E-cadherin antibody. Ubiquitinated E-cadherin was analyzed by western blot with a K48/K63-specific antibody (*right*). (JPG 1036 kb)

Additional file 8: **Figure S4.** E-cadherin loss was sufficient for EMT. A, H522 cells stably transfected with a lentiviral control shRNA or E-cadherin shRNA (E-cad KD) were seeded overnight. E-cadherin (E-cad), Vimentin (Vim), and β-actin in TCLs were detected by western blot. β-catenin was detected in the H522 cell nuclear extract. B, EMT morphological changes and micrometastatic incidences in H522 cells transfected with control shRNA and E-cadherin shRNA. Scale bars, 50 μm. (E-cad KD, *χ*^*2*^ test, *, *P* < 0.05). (JPG 225 kb)

Additional file 9: **Figure S5.** Frz8-Dvl3 interaction. A, Schematic representation of reporter plasmids containing full-length Frizzled 8 (Frz8 WT) and truncated Frz8 (Frz8-CRD). B, Frz8-knockdown A549 cells stably transfected with Frz8 WT or Frz8-CRD via adenovirus were seeded overnight. The TCLs were subjected to IP using anti-E-cadherin and anti-HA antibodies. Ubiquitinated E-cadherin, RNF43, and HA were detected by western blot (*upper and middle blot*). E-cadherin and β-actin in the TCLs were detected by western blot (*lower blot*). C, A549 cells stably transfected with the control vector or Dishevelled 3 (Dvl3) via adenovirus were seeded overnight. The TCLs were subjected to immunoprecipitation using an anti-E-cadherin antibody. Ubiquitinated E-cadherin, E-cadherin, and RNF43 were detected by western blot. D, A549 cells stably transfected with the control vector or Dvl3 via lentivirus were seeded overnight. The TCLs were subjected to IP using anti-Frz8. Ubiquitinated Frz8, Dvl3, and Frz8 were detected by western blot. E, A549 cells stably transfected with the control or ZNRF3 via adenovirus were seeded overnight. The TCLs were subjected to IP using an anti-E-cadherin antibody. Ubiquitinated E-cadherin was detected by western blot with an anti-ubiquitin antibody (*upper blot*). E-cadherin, Vimentin, ZNRF3, and β-actin in the TCLs were detected by western blot (*middle blot*). β-catenin was detected in the nuclear extract of A549 cells (*lower blot*). F, EMT morphological changes and metastatic incidences in A549 cells stably transfected with the lentiviral control or ZNRF3. Scale bars, 50 μm. (*χ*^*2*^ test, *, *P* < 0.05). (JPG 1301 kb)

Additional file 10: **Figure S6.** Schematic illustration of the RNF43-initiated EMT signaling pathway. (JPG 335 kb)

RETRACTED

## Data Availability

The datasets used and/or analyzed in this study are available from the corresponding author upon reasonable request.

## Abbreviations

AJCC: American Joint Committee on Cancer
ATCC: American Type Culture Collection
BSA: Bovine serum albumin
Casp8: Caspase-8
CH2: Cadherin homology 2
ChIP: Chromatin immunoprecipitation
CNBr: Cyanogen bromide
CRD: Cysteine-rich domain
Dvl: Dishevelled
E-cad: E-cadherin
EMT: Epithelial-mesenchymal transition
Frz: Frizzled
GST-SH2: Glutathione S-transferase-SH2
HE: Hematoxylin-eosin
LGR: Leucine-rich repeat-containing G protein-coupled receptor
MDCK: Madin Darby canine kidney
NSCLC: Non-small cell lung cancer
OS: Overall survival
PA: Protease domain
PVDF: Polyvinylidene difluoride
p-β-catenin: Phospho-β-catenin
RIPA: Radioimmunoprecipitation
RNF43: RING finger protein 43
RSPO: R-spondin
RT-PCR: Reverse transcription-polymerase chain reaction
SDS-PAGE: SDS-polyacrylamide gels
shRNA: Short hairpin RNA
STR: Short tandem repeat
TBST: Tris-buffered saline Tween-20
TCF/LEF: T-cell factor/lymphoid enhancer factor
TCL: Total cell lysate
TFA: Trifluoroacetic acid
Tyr: Tyrosine
Vim: Vimentin
WRE: Wnt-responsive element
WT: Wild-type
